# Phytochemical Classification of Medicinal Plants Used in the Treatment of Kidney Disease Based on Traditional Persian Medicine

**DOI:** 10.1155/2022/8022599

**Published:** 2022-07-31

**Authors:** Fatemeh Rabizadeh, Maryam Sadat Mirian, Rahele Doosti, Roya Kiani-Anbouhi, Elahe Eftekhari

**Affiliations:** ^1^Farzanegan Campus, Semnan University, Semnan, Iran; ^2^Central Herbarium of Tehran University, College of Science, University of Tehran, Tehran, Iran; ^3^Faculty of Chemistry, Shahrood University of Technology, Shahrood, Iran; ^4^Department of Chemistry, Faculty of Sciences, Imam Khomeini International University, Qazvin, Iran; ^5^Department of Biology, Science and Research Branch, Islamic Azad University, Tehran, Iran

## Abstract

**Methods:**

This review was focused on studying the various secondary metabolites in model plants of Iranian herbal medicine known as treatment of kidney diseases in traditional Persian medicine textbooks including Makhzan-ol-Advieh, The Canon of Medicine, and Taghvim al-Abdan fi Tadbir al-Ensan.

**Results:**

Secondary metabolites of 94 medical plants belonging to 42 families were reported with their scientific and family name.

**Conclusion:**

Although herbal medicines are gaining rapid popularity among people and the pharmaceutical industry, the understandings of the phytochemical and therapeutic properties of medicinal plant are important for developing effective nephroprotective medicines. Therefore, the relationship between traditional uses and biological properties should be clearly verified through further studies.

## 1. Introduction

Since ancient times, natural products, such as parts of plants, animals, and microbes have been utilized in medicine to treat diseases. According to fossil records, human usage of plants as remedies may be dated back at least 60,000 years [1]. Over the past decade, an increasing attention has been focused on the effect of medicinal plants. Traditional herbs from different habitats and geographical locations can be considered as a new strategy for the treatment of injuries and protection against infections.

The kidney, as a vital organ, controls water balance, maintains electrolyte concentrations, removes nitrogenous waste products, and regulates blood pressure in the body [2]. The kidney is very susceptible to damage and injury and it might lose its function and cannot act as it should. Kidney diseases can be made up from inherited mutations [3] and chronic injuries, such as diabetes [4] and inflammatory diseases [5]. Moreover, the most famous renal failure known as kidney stone is appeared by abnormal accumulation of crystalline substances such as calcium. Typically, surgery of kidney stone causes to appear serious difficulties such as urinary tract obstruction, abnormal urine metabolism, and hydronephrosis [6]. This critical organ also goes through the processes of anatomical and physiological changes by aging, obesity, and hypertension. Moreover, a greater number of individuals have been diagnosed with chronic renal failure, which the body is unable to maintain metabolic, fluid, and electrolyte balance, resulting in a retention of urea and other nitrogenous wastes in the blood [7, 8]. The kidney is also remarkably prone to drug-induced toxicity due to exposure to the largest proportion of circulating chemicals and drugs [9]. Despite remarkable advances in diagnostic and treatment techniques of kidney diseases, the prevalence of renal dysfunction has been increasing in recent years. Interestingly, numerous experimental studies have revealed that herbal medicine has a beneficial effect on improving kidney function.

Epidemiological evidence suggests that natural bioactive substances play an essential role in the treatment and control of modern diseases [10]. Natural products, which have evolved over millions of years, have a distinct chemical diversity and result in a wide range of biological activities and drug-like qualities [1]. Plants produce constitutive metabolites known as phytochemicals which play a critical role in their survival and proper function. These chemical components not only protect plants from competitors, pathogens, or predators but also control the growth along with regulating the pollination, fertilization, and the rhizosphere environment [11]. Phytochemicals can be found in various parts of plant, including stems, leaves, roots, seeds, fruits, and flowers. However, many phytochemicals, notably color compounds, are found in high concentrations in the outer layers of plant tissues [12]. Previous investigations have reported that phytochemicals lead to reduction in the risk of some diseases such as coronary heart, diabetes, liver disorders, high blood pressure, as well as reducing the synthesis or absorption of cholesterol [13].

Phytochemicals are classified as primary and secondary metabolites, based on their function in plant metabolism. Primary metabolites are necessary for plant life and include carbohydrates, amino acids, proteins, lipids, purines, and pyrimidines of nucleic acids. On the contrary, secondary metabolites are the remaining plant chemicals produced by the cells through metabolic pathways derived from the primary metabolic pathways [14, 15]. These chemical components have been described as an antiviral, antifungal, and antibiotic, which are responsible for protecting plants from pathogens. Additionally, they are critical UV absorbing chemical factors, preventing severe leaf damage from the light [16]. Due to their great biological activities, plant secondary metabolites have been exerted for centuries in traditional medicine and the medicinal effects of the plants come from these molecules [17]. Moreover, various tissues and organs of medicinal plants could have peculiar medicinal properties at specific developmental phases [18]. These days, they are associated with valuable industries such as pharmaceutics, cosmetics, and fine chemicals [19].

Secondary metabolites in plants are classified into three main groups based on their biosynthetic pathway; (a) nitrogen-containing compounds such as alkaloids, glucosinolates, and cyanogenic glycosides, (b) phenolic compounds such as phenylpropanoids and flavonoids, and (c) terpenes [17, 20]. Alkaloids are a class of nitrogen-containing compounds produced in plants in response to biotic or abiotic environment which endows alkaloids to possess remarkable biological activities and structure diversity [21, 22]. Cyanogenic glycosides are amino acid-derived plant components found in more than 2500 plant species and are widely distributed among 100 families of flowering plants [23, 24]. The toxicity of cyanogenic glycoside derivatives is based on the release of hydrogen cyanide [25]. Glucosinolates contain sulfur and nitrogen produced in some plants and are chemically stable under normal conditions [26]. The nonprotein amino acids are structurally similar to protein amino acids and particularly participate in plant defense against stress and act as essential mediators in response to abiotic factors [27]. Amines as low molecular weight are nitrogenous compounds which are naturally present in plants and are responsible for many biological effects such as acting as important precursors of hormones [28]. Phenolic components are derived from shikimate, pentose phosphate, and phenylpropanoid pathways in plants and have an aromatic ring with one or more hydroxyl groups [29, 30]. Glycosides are usually organic molecules isolated from plant sources and consist of one or more sugars incorporated with phenol, alcohol, or a complex molecule such as a steroid nucleus [31]. Terpenoids are the most abundant group of plant secondary metabolites typically produced in flowers, vegetative tissues, and, roots [32]. They show a broad range of biological activities which result in lower total cholesterol, triglycerides, or LDL‐cholesterol, as well as blood pressure [33]. A variety of toxic proteins are expressed in plants and act as resistance factors against plant pathogens and herbivores. Most of toxic proteins accumulate in the vulnerable parts of the plant, such as vegetative storage tissues and seeds [34]. Carbohydrates are produced through photosynthesis in plants and are a crucial source of energy and carbon skeletons for organic compounds and storage components. In addition, they act as signaling molecules as same as hormones [35, 36]. 6, 9-polyunsaturated fatty acids are produced by plants and are essential to the human diet. These components are of importance increasingly as raw materials for industry [37]. Organic acids are intermediate or end products in various fundamental pathways in plant metabolism and catabolism [38].

The effect of medicinal plant utilizes is global and it has been expanding in numerous countries over the world [39]. Importantly, traditional Persian medicine as a source of alternative therapies has become popular over Iran and some countries globally. Iranian herbal medicine consists of natural compounds with complex active ingredients that cause valuable effects. Traditional Persian medicine has been widely used in treating kidney diseases due to its safety and economic advantages. Because of advances in modern technology, it is now possible to assess the pharmacology and mechanisms related to function of many Iranian herbs. A wide range of these medicinal plants has been studied to further apply of plants' function for agriculture, medicine, and chemical industries. This review was focused on studying the various secondary metabolites in model plants of traditional Persian medicine which they are known as a treatment of kidney diseases and injuries in traditional Persian medicine textbooks. We have given the review based on the most important clinical and pharmaceutical traditional Persian medicine textbooks, including Makhzan-ol-Advieh by Aqili (18^th^ century), The Canon of Medicine by Avicenna (10^th^ and 11^th^ centuries), and Taghvim al-Abdan fi Tadbir al-Ensan (11^th^ century). In this review, we investigated nitrogen-containing compounds including glucosinolates, alkaloids, cyanogenic glycosides, nonprotein amino acids, amines, and toxic proteins. Additionally, compounds including phenolic components, terpenoids, glycosides, carbohydrates, fatty acids, and organic acids were considered as non-nitrogen-containing components of medical plants.

## 2. Methods

First, we have gathered all information of medical plants which were responsible for the treatment of kidney diseases and introduced in Makhzan-ol-Advieh, The Canon of Medicine, and Taghvim al-Abdan fi Tadbir al-Ensan. Then, we have classified them into their scientific name and discussed their phytochemical composition in the next topic. We have collected reports from scientific articles from journals indexed online in PubMed, Science Direct, and Medline. The main findings are summarized in figures and a table.

## 3. Result

In the current review, a total of 94 medical plant species belonging to 42 families have been reported to treat kidney diseases in traditional Persian medicine textbooks specifically.  Table 1 shows bioactive and secondary metabolites of medicinal plants of traditional Persian medicine with their scientific and family name. Among them, *Apiaceae* (11 species), *Alliaceae* (7 species each), *Pinaceae*, *Fabaceae* (6 species each), *Lamiaceae*, *Malvaceae*, and *Asteraceae* (5 species) were the dominant families.

Figure 1 represents the ratio of two groups of bioactive components in the medical plant of this study. It is shown that the phytochemical components without nitrogen are the major part of these plants (82%) compared to the nitrogen containing component (18%).

As can be seen in Figure 2, most of the present medicinal plants contained terpenoids (63%) with considerable effects on the treatment of renal failure. 53% of mentioned plants possessed phenolic components. Moreover, organic acids, fatty acids, and glycosides were observed in 26%, 23%, and 22% of medicinal plants, respectively. Among the nitrogen-containing components, alkaloids were seen in 17% of plants and toxic proteins, nonprotein amino acids, amines, cyanogenic glycosides, and glucosinolates were demonstrated in 13%, 8%, 4%, 2%, and 1% of plants, respectively.

## 4. Discussion

Plants play an essential role in primary health care and treatment of diseases and disorders in traditional medicine. Kidney disorders and urinary infections are common in people over the world and a large number of research works has been done to overcome these challenges. Medicinal plants offer an attractive source for improving kidney function and treating the symptoms of renal disorders. Herein, we have systematically summarized the secondary metabolites of the medical plants introduced in traditional Persian medicine books.

Several studies have shown the kidney treatment properties of some plants presented in the current review on the folk and traditional medicines of the Mediterranean, China, Bulgaria, and Turkey. In Bulgarian traditional and folk medicine, *Arum maculatum* tuber has been shown to be widely used in cases of kidney stones [137]. Furthermore, aerial parts of *Petroselinum crispum* impact kidney stones by consuming a decoction of fresh roots as tea in Turkish folk medicine [138]. In European herbal medicine, *Cichorium pumilum* is known helpful in cleaning the body and stimulating the eliminative process both via intestines and kidneys [139]. The traditional medicine in Algeria believes that *Pinus halepensis* act as medical plants for healing stomachaches and kidney inflammations [140]. *Alisma plantago* L. ameliorates hypertension and renal injury based on traditional Chinese medicine [141].

Although these herbal medicines are popular in folk culture, the understandings of the phytochemical and the mode of action of based-plant medicines are of great importance for the development of safe and effective nephroprotective drugs. Over the past years, numerous studies have been performed on some of these traditional medicine plants to investigate their effect on kidney dysfunction. According to the previous papers, *Cocos nucifera* L. was a urinary antiseptic and coconut water seemed to have protective effects and treated kidney and urethral stones effectively [142, 143]. Aloe vera leaf gel extract showed improvement in the mild damage caused by type2 diabetes on kidney tissue [144]. Aqueous and ethanolic extract powders of dried *Syzygium aromaticum* buds include adequate gallic acids which are one of the considerable compounds of phenolic. It was shown to have a strong antioxidant impact of gallic acid on kidney dysfunction in rats [145]. *Equisetum arvense* L. with traces of alkaloids, flavonoids, triterpenoids, phytosterols is the most popular species from the Equisetum genus whose diuretic effects were confirmed in animal models and clinical trials [84]. Camphor is found in roots and stem of the *Cinnamomum camphora* and is produced for health, medical, and industrial applications. Camphor treatment of diabetic rats reduced the oxidative stress markers in the liver and kidney tissues compared to control rats [146]. It was observed that treatment with *Allium porrum* L. extract decreased the number of crystals in kidney sections, and creatinine levels in treated animals in comparison with the control group. It suggested that the plant could be an excellent candidate to inhibit the formation of calcium oxalate crystals in the kidney [147].

Due to the active ingredients and active flavonoids of *Pistacia vera* L., the hydroalcoholic extract was effective on urinary tract (kidney and bladder) disorders by the reducing inflammation and oxidative stress in the kidney. Pistachio extract enhanced creatinine clearance and reduced the urine volume, urine glucose, serum creatinine, blood urea nitrogen levels, and histopathological scores in all doses; however, the highest change was seen at dose of 100 mg/kg [148]. The impact of the extract of *Carum copticum* seeds was investigated on the urinary stones of 350 patients. 100%, 53%, and 31.25%, of calcium oxalate, calcium oxalate/uric acid, and calcium-oxalate/hydroxyapatite stones, respectively, were treated with the extract [149]. Phytochemical screening showed that *Capparis spinosa* seed extracts consist of high level of phenolic compounds with individual molecules with high nephroprotective and hepatoprotective activity. Histopathological observation confirmed that pretreatment with extract of *C*. *spinosa* improved the damages detected in the kidney [150]. A paper reported that the dose of 200 mg/kg and 400 mg/kg of methanolic extract of *Laurus nobilis* preserved the functional capacity of the kidney against paracetamol toxicity in treated rat [151]. It was reported that the administration of *Malva sylvestris* extract not only significantly protected against lithium-induced oxidative damage, histopathological damage, and biochemical changes but also decreased the abnormal features detected in kidney slices of poisoned rats due to the presence of phenolic acids and flavonoids [152, 153]. The *Morus alba* L. methanolic extract in different mice organs improved the oxidative stress in kidney and consequently, renal functions were modulated. It suggested that the presence of the phenolic groups such as quercetin and naringenin in *M. alba* could be responsible for OH radical scavenging activity [154]. Supplementing with *Sesamum indicum* L. oil showed a significant reduction in ALP activities in the kidney with no corresponding increase in the serum, thus suggesting that the benniseed oil appears to attenuate the effect the hypercholesterolemic diet on the kidney [155]. In treatment of calcium oxalate urolithiasis in rats with *Piper cubeba* L. fruit extract, urinary crystals and histopathological derangement were improved at the doses 35 mg/kg and 60 mg/kg through significant decrease in urinary calcium after 14 days [156]. *Oryza sativa* L., as a rich source of anthocyanin, was investigated in renal function in obese rats. It was observed to show a reduction in renal injury by the attenuation of either oxidative stress, or apoptosis of renal cells [157].

A paper indicated that *Zizyphus jujuba* aqueous extract at a concentration of 500 mg/kg had a therapeutic role in reducing nephrotoxicity induced by ibuprofen that is a nonsteroidal anti-inflammatory drug and relieves pain and swelling [158]. The *Citrus aurantium* L. extract at a dose of 200 mg/kg was treated for a period of 21 days against gentamicin-induced renal damage. According to the results, *C*. *aurantium* L. extracts successfully protected renal damage associated with gentamicin due to its flavonoid contents and antioxidant properties [159]. Hydroalcoholic extract of *Physalis alkekengi* L. at a dose of 420 mg/kg was investigated for its nephroprotective activity against cisplatin-induced acute renal injury in rats of either sex for 10 days. The results showed a significant reduction in the elevated blood urea, serum creatinine, and uric acid and also normalized the histopathological changes [160]. Additionally, the biochemical and histopathological results clarified the role of phenolic-rich *Vitis vinifera* L. in improving the toxicity of CCl_4_ in the kidney of rats by suppressing the ROS/NF-*κ*B signaling pathway [161].

Ideally, more investigations on the chemical and pharmacological activities of these medicinal plants are needed to discover their mechanisms and to define the metabolites responsible for their activities. Furthermore, promising chemical compounds should be extracted to find their effects on the treatment of kidney failure and the relationship between biological features and traditional uses should be clearly verified through further studies.

## Figures and Tables

**Figure 1:** The ratio of phytochemical components of the medicinal plants studied in the current review.

**Figure 2:** Percentage of the medicinal plants containing secondary metabolites studied in the current review.

**Table 1:** Secondary metabolites of medicinal plants are used to treat kidney diseases according to traditional Persian medicine.

No.	Scientific name	Family name	Glycoside	Organic acid	Carbohydrate	Fatty acid	Phenolic	Terpenoid	Toxic protein	Glucosinolate	Cyanogenic glycoside	Amine	Non-protein amino acid	Alkaloid	References
1	*Alisma plantago* L.	*Alismaceae*					Ferulic acid, Rosmarinic acid	Triterpenes, diterpenes, sesquiterpenes							[40]
2	*Allium ampeloprasum* L.	*Alliaceae*						Pinene, beta-pinene		Dimethyl tetrasulphide					[41]
3	*Allium ascalonicum* L. (*Allium minutiflorum*)	*Alliaceae*	*β*-D-glucopyranoside]					Furostanol saponins							[42]
4	*Allium cepa* L.	*Alliaceae*	Quercetin glucosides	Formic acid				Humulaneand phytosterols	Fluorescent protein						[43]
5	*Allium porrum* L.	*Alliaceae*						Sapogenin							[44]
6	*Allium roseum* L.	*Alliaceae*			Tetradecane	Hexadecanoic acid	Tricosane								[45]
7	*Allium ursinum* L.	*Alliaceae*					Kaempferol		Lectins						[46]
8	*Allium vineale* L. (Allium vegetable)	*Alliaceae*							*β*-chlorogeni						[47]
9	*Pistacia lentiscus* var. Chia	*Anacardiaceae*			Limonene		Trans-pinocarveol	Α-pinene, *α*-terpinolene							[48, 49]
10	*Pistacia lentiscus* L.	*Anacardiaceae*		Cadinene	Oleanonic acid		Phytol, *α*-cadinol	*α*-terpineol							[50]
11	*Pistacia vera* L.	*Anacardiaceae*				Palmitic acid	Pinocarveol								[51]
12	*Anethum graveolens* L.	*Apiaceae*						*β*-pinene, p-cymene, limonene							[52]
13	*Apium graveolens* L.	*Apiaceae*	Sucrose				Geraniol						*β*-amyloid		[53]
14	*Carum bulbocastanum*—(Boiss.) B. Fedtsch.	*Apiaceae*			Dillapiole	*β*-Germacrene-									[54]
15	*Carum carvi* L.	*Apiaceae*				Benzenedicarboxylic acid		Limonene, carvone							[55]
16	*Carum copticum* L.	*Apiaceae*					Thymol	*β*-pinene, *α*-pinene							[56, 57]
17	F*erula assa- foetida* L.	*Apiaceae*			P-Cymene		Thymol	*α*-pinene, phellandrene							[58]
18	*Ferula narthex*	*Apiaceae*						Coumarins							[59]
19	*Lagoecia cuminoides* L.	*Apiaceae*						A-pinene, myrcene, limonene							[60]
20	*Petroselinum crispum*	*Apiaceae*		1,2 benzene-dicarbonic acid				Α-pinen, *β*-phellandrene							[61, 62]
21	*Seseli tortuosum* L. (Seseli libanotis)	*Apiaceae*					Coumarin	Myrcene							[63]
22	*Sium latifolium* L.	*Apiaceae*						*α*-thujene, *α*-pinene							[64]
23	*Arum italicum* L.	*Araceae*					Guaiacylglycerol-*β*-coniferyl				8-O-4′-neolignan glucoside				[65]
24	*Arum maculatum* L.	*Araceae*						*α*-pinene, *β*-pinene, terpinolene					Indole		[66]
25	*Colocasia antiquorum* (Colocasia esculenta)	*Araceae*				10-octadecenoic acid							Trypsin		[67]
26	*Cocos nucifera* L.	*Arecaceae*	Sucrose, glucose, fructose	Ascorbic acid	Carbohydrate				Tryptophan				Alanine*β*-Alanine, Aspartic acid	Thiamin	[68]
27	*Asarum europaeum* L.	*Aristolochiaceae*					*α*-Asarone, *β*-Asarone								[69]
28	*Asparagus adscendens*	*Asparagaceae*					Spirostanosides				*β*-D-glucopyranosyl]-(25S)-spirostan-5-en-3*β*-ol				[70]
29	*Asparagus officinalis* L.	*Asparagaceae*					Capsanthin, Violaxanthin								[71]
30	*Asparagus racemosus*	*Asparagaceae*				n-Hexadecanic acid, Oleic acid									[72]
31	*Aloe vera* L.	*Asphodelaceae*	Glucomannan	Oxalic acid		Tridecanoic acid	Anthraquinone/Phytol								[73]
32	*Artemisia abrotonon* L. (Artemisia abyssinica) (Artemisia ketone) (Artemisia annua)	*Asteraceae*					1,8-cineole	Methyl eugenol, camphor	Total protein					Alkaloids	[74]
33	*Artemisia montana* (Artemisia ketone, Artemisia annua)	*Asteraceae*		Ascorbic acid			Quercetin	Camphor							[75]
34	*Chrysanthemum indicum* L.	*Asteraceae*		Naphthaleneboronic acid	*β*-Myrcene		Bornyl acetate	Camphor							[76]
35	*Cichorium intybus* L.	*Asteraceae*	Glycosides			Fatty acids	Lactucin, 8-deoxylactucin	Lactupicrin						Alkaloids	[77]
36	*Cichorium pumilum*	*Asteraceae*	Lactucin				Anthocyanins	Anthocyanins							[78]
37	*Capparis decidua* (Capparis cartilaginea, Capparis deserti)	*Capparidaceae*	Butyl isothiocyanate	Ascorbic acid	Cellulose				Isothiocyanate					Alkaloids	[79]
38	*Capparis spinosa* L. (Capparis sicula)	*Capparidaceae*	Capparisine	Protocatechuric acid		(z,z)-9,12-octadecadienoic acid	Furfural, Bis(5-for-mylfurfuryl) ether							Capparisine	[80]
39	*Cucumis colocynthis* L.	*Cucurbitaceae*	Cucurbitacin glucosides				Isosaponarin								[81]
40	*Cyperus longus* L.	*Cyperaceae*						*α*-longipinene							[82]
41	*Cyperus rotundus L.*	*Cyperaceae*			Myrcene		Isocurcumenol	Α-pinene, P-cymene						Alkaloids	[83]
42	*Equisetum arvense L.*	*Equisetaceae*					Hexahydrofarnesyl acetone, Thymol								[84]
43	*Acacia catechu (L.)* *(Acacia Concinna)*	*Fabaceae*		Malic acid			Saponins							Alkaloids	[85]
44	*Alhagi mannifera* *(Alhagi maorurum)* *(Alhagi pseudalhagi)*	*Fabaceae*		Saliylic acidvanillic acid			Quercetin							Salsolidine	[86]
45	*Glycryrrhiza glabra L.*	*Fabaceae*	Pectin				Flavonoids	Triterpene							[87]
46	*Phaseolus vulgaris L.* *(Phaseolus aureus)*	*Fabaceae*		Trichloroacetic acid					L-tryptophannone					N-acetyl mannosamine	[88]
47	*Vigna reflexo-pilosa* *(Vigna radiata)*	*Fabaceae*				Oleic acid	Galactosylononitol								[89]
48	*Vigna unguiculata*	*Fabaceae*					Sterols	Triterpene							[90]
49	*Ajuga chamaepitys (L.)* *(Ajuga. Reptans)*	*Lamiaceae*	(*α*-1,6-galactosyl sucrose)		Carbohydrate		Iridoid								[91]
50	*Ajuga iva L.* *(Ajuga orientalis)* *(Ajuga bracteosa)*	*Lamiaceae*					Linalool Methyl salicylate	Limonene							[92]
51	*Melissa officinalis L.*	*Lamiaceae*	Epigallocatechin-3-gallate	Rosmarinic acid	Β-carotene		Anthocyanidin, Curcumin	Citral						Caffeine, Nicotine	[93]
52	*Origanum majorana L.*	*Lamiaceae*					4-terpineol	Sabinene							[94]
53	*Teucrium chamaedrys L.*	*Lamiaceae*			Bicyclo [4.4.0] dec-1-ene		2-Pentadecanone	*α*-pinene, *β*-pinen							[95]
54	*Cinnamomum bejolghota*	*Lauraceae*						Terpenes				Phenylpropanoids			[96]
55	*Cinnamomum camphora*	*Lauraceae*			Hexadecy			Α-thujene, *α*-pinene, camphene							[97]
56	*Laurus nobilis L.*	*Lauraceous*				Lauric acid, Myristic acid	Terpinenol	Camphene sabinene, myrcene							[98]
57	*Hyacinthus orientalis*	*Liliaceae*	Anthocyanin 3,5-diglucosides	P-cis-coumaric acid, caffeic acid, malonic acid			Delphinidin								[99]
58	*Linum catharticum L.*	*Linaceae*				Octadecanoic acid						(2-hydroxyethyl)amide			[100]
59	*Linum usitatissimum L.*	*Linaceae*		Vanillic acid		*α*-linolenic acid							Aspartine, Threonine		[101]
60	*Malva sp.* *(Malva mauritiana)*	*Malvaceae*	D-glucose												[102]
61	*Althaea sp.*	*Malvaceae*				Stearic acids		Trenoids							[103]
62	*Gossypium herbaceum L.*	*Malvaceae*				Linoleic acid	*β*-bisabolol	Tetrahydrolinaloo							[104]
63	*Malva parviflora L.*	*Malvaceae*			Cyclopropene										[105]
64	*Malva sylvestris* L.	*Malvaceae*				*α*-linolenic acid	Quercetin								[106]
65	*Ficus sycomorus L.*	*Moraceae*		3-acetyl-citric acid			Ethyl-4-methyltetrahydrofuran-3-ol								[107]
66	*Morus alba* L.	*Moraceae*	Cyanidin-3-glucoside, cyanidin-3-glucosylrhamnoside				Apigenin								[108]
67	*Musa* sp.	*Musaceae*		Ascorbic acid, vitamin A				*β*-carotene, *α*-carotene							[109]
68	*Syzygium aromaticum* (L.)	*Myrtaceae*		Hexadecanoic acid			Eugenol,	Thymol, caryophyllene oxide	Proteins p53, protein bcl-2						[110]
69	*Sesamum indicum* L.	*Pedaliaceae*	Sesaminol glucosides				1-hydroxypinoresinol, antioxidant lignans		*α*-Globulin						[111]
70	*Pinus cembera* L. *Pinus cembra* L.	*Pinaceae*						Limonene, *β*-phellandrene, *α*-pinene							[112]
71	P*inus eldarica*	*Pinaceae*	Flavonoids				Proanthocyanins, Flavonols								[113]
72	*Pinus halepensis*	*Pinaceae*			Carbohydrate	Myristic, oleic and linoleic acids		Terpenes, *α*-*β*-pinene, limonene	Protein						[114]
73	*Pinus nigra*	*Pinaceae*						*α*-pinene							[115]
74	Pinus pinea L.	*Pinaceae*				Fatty acid		Monoterpene, *β*-pinene							[116]
75	*Pinus sylvestris* L.	*Pinaceae*		Naphthaleneacetic acid	Sucrose			Monoterpene, *α*-pinene				Benzyladenine	Phenylalanine		[117]
76	*Piper cubeba* L.	*Piperaceae*						Linalool, caryophyllene							[118]
77	*Piper nigrum* L.	*Piperaceae*		Carboxylic acids, 2,4 tetradecadienoic acid		Tetracosanoic acid	Anthraquinones	Cadinene, caryophyllene						Piperine, lkaloids	[119]
78	*Oryza sativa* L.	*Poaceae*			Oligosaccharide				Glycoproteins, *α*1-acid glycoprotein				Tryptophan	Indole-alkaloid glucoside	[120]
79	*Polyporus officinalis*	*Polyporaceae*		Methyl jasmonate		Hexacosanoic acids, pentadecanoic acid									[121]
80	Anagallis arvensis L.	*Primulaceae*	Saponins												[122]
81	*Zizyphus jujuba* (Zizyphi Spinosi semen)	*Rhamnaceae*	Saponins												[123]
82	*Prunus avium* L.	*Rosaceous*		Phenolic acid, protocatechuic acid			Tannic acid, protocatechuic acid	Thymol, carvacrol							[124]
83	*Rubus fruticosus* L.	*Rosaceous*						Lanceol							[125]
84	*Nauclea* sp.	*Rubiaceae*		9,12-octadecadienoic acid, 2-oxopentanedioic acid	Carbohydrates	17-octadecynoic acid, ethyl ester	Phenolics, 2-methoxy-4-vinylphenol	Phytol, terpenoids						Alkaloids	[126]
85	*Citrus aurantium* L.	*Rutaceae*						Geraniol, a-terpineol				Methyl anthranilate			[127]
86	*Physalis alkekengi* L.	*Solanaceae*	Glycosides, physanosides				Luteolin	6S,9R)-roseoside, (6S,9S)-roseoside, citroside A						Alkaloids, hyoscyamine	[128]
87	*Styrax officinalis* L.	*Styracaceae*					Eugenol	Terpenoids, linalool							[129]
88	*Aquilaria malaccensis* (*Aquilegia vulgaris* L., *Aquilegia canadensis* L., *Aquilegia chrysantha*, *Aquilegia glandulosa*)	*Thymelaeaceae*				Fatty acid		Caryophyllene oxide							[130]
89	*Trapa natans* L.	*Trapaceae*						(all E)-squalene							[131]
90	*Nardostachys jatamansi*	*Valerianaceae*		Nardin			Coumarins	Sesquiterpenes						Alkaloids	[132]
91	*Valeriana celtica* L *Valeriana officinalis* L. *Valeriana wallichii* (*Valeriana italica*, Valeriana tuberosa(3))	*Valerianaceae*		3-Methyl valeric acid		Isovaleric acid, tetradecanoic acid	Lignans, caffeic acid derivatives	Valerenic acid, sesquiterpene, monoterpenoids					Amino acids	Alkaloids	[133]
92	*Viola odorata* L. (Viola etrusca)	*Violaceae*						*α*-Pinen, xamphene							[134]
93	*Viola tricolor* L.	*Violaceae*			Mucilages			Saponins, carotenoids							[135]
94	*Vitis vinifera* L.	*Vitaceae*						Farnesene							[136]
